The article "Intensity-Modulated Radiation Therapy Optimization for Acceptable and Remaining-One Unacceptable Dose-Volume and Mean-Dose Constraint Planning" was published in 2020. Journal: Comput Math Methods Med.

# Intensity-Modulated Radiation Therapy Optimization for Acceptable and Remaining-One Unacceptable Dose-Volume and Mean-Dose Constraint Planning

**DOI:** 10.1155/2020/3096067

**Published:** 2020-09-03

**Authors:** Ryosei Nakada, Omar M. Abou Al-Ola, Tetsuya Yoshinaga

**Affiliations:** ^1^Graduate School of Health Sciences, Tokushima University, 3-18-15 Kuramoto, Tokushima 770-8509, Japan; ^2^Faculty of Science, Tanta University, El-Giesh St., Tanta, Gharbia 31527, Egypt; ^3^Institute of Biomedical Sciences, Tokushima University, 3-18-15 Kuramoto, Tokushima 770-8509, Japan

## Abstract

We give a novel approach for obtaining an intensity-modulated radiation therapy (IMRT) optimization solution based on the idea of continuous dynamical methods. The proposed method, which is an iterative algorithm derived from the discretization of a continuous-time dynamical system, can handle not only dose-volume but also mean-dose constraints directly in IMRT treatment planning. A theoretical proof for the convergence to an equilibrium corresponding to the desired IMRT planning is given by using the Lyapunov stability theorem. By introducing the concept of “acceptable,” which means the existence of a nonempty set of beam weights satisfying the given dose-volume and mean-dose constraints, and by using the proposed method for an acceptable IMRT planning, one can resolve the issue that the objective and evaluation are different in the conventional planning process. Moreover, in the case where the target planning is totally unacceptable and partly acceptable except for one group of dose constraints, we give a procedure that enables us to obtain a nearly optimal solution close to the desired solution for unacceptable planning. The performance of the proposed approach for an acceptable or unacceptable planning is confirmed through numerical experiments simulating a clinical setup.

## 1. Introduction

Intensity-modulated radiation therapy (IMRT) [1, 2], which is a type of external beam radiotherapy, is an advanced radiotherapy technique used to reduce the amount of normal tissue exposed to radiation in the treatment area. It also improves the ability to conform to the volume of treatment applied to concave tumor forms. The radiation delivery pattern is determined using computerized applications designed to perform optimization and therapeutic simulations. The radiation dose is adjusted by modifying the intensity of the beam in accordance with the shape of the tumor. The intensity of the radiation dose is raised near the tumor but is reduced or zero among adjacent normal tissues, i.e., a radiation field with a nonuniform (i.e., modulated) intensity is delivered. Compared with conventional nonmodulated radiotherapy techniques with beams of uniform intensity, IMRT leads to better tumor targeting and mitigation of side effects, which may increase the chance of curing the patient. Furthermore, recently, volumetric modulated arc therapy (VMAT) has been adopted in clinical practice. One of the features of VMAT is that it performs IMRT while rotating the specific range of gantry, which increases the flexibility of generating a theoretically highly conformal treatment plan [3–5].

The calculation of nonuniform intensities based on the dose prescription in the planning target volume (PTV) and the neighboring critical or sensitive organs, called organs at risk (OARs), is called inverse planning. IMRT inverse treatment planning uses optimization techniques, with the objective function measuring the quality of a treatment plan, to form the dose distribution with the ability to generate concave dose distributions and provide a specific spacing for the sensitive normal structures. The dose-volume constraint (DVC) expressed as an inequality condition with a set of a volume percentage and prescription dose applied to a PTV or OAR is evaluated on specific, predefined subvolumes of the organ and restricts the relative volume of a structure that receives more or less than a particular threshold. The use of DVCs is a normal way to determine the objective and has been the standard way of evaluating the treatment in practice; however, they are generally handled in limited ways in current optimization algorithms. Namely, because the inequality with percentages is difficult to treat as an objective function in optimization, the conventional methods are mostly constructed by using gradient techniques such as Newton's method and the conjugate gradient method of minimizing dose-based and biology-based objective functions [6–11], and therefore, one expects to obtain a feasible solution violating the DVCs in a minimal way. Due to the difference between the *objective* for optimization and the *evaluation* for the planning result, a trial-and-error approach was required in the DVC-based planning process [12], more specifically as follows: When the given DVC is too tight, planners cannot easily obtain the optimal solution and the goal of treatment planning is not achieved. On the other hand, when the given DVC is too loose, planners can obtain the optimal solution, but there is room for improvement in IMRT treatment planning. In order to obtain an achievable and high-quality IMRT treatment planning, planners are required to find optimal DVC settings for each clinical case. As a result, it takes a lot of time to perform trial and error. Furthermore, the quality of the treatment planning varies from planner to planner [13]; a useful approach is required that supports planners in obtaining high-quality treatment planning in a short time. For example, on the hardware side, there is an approach to perform faster calculations utilizing a graphics processing unit (GPU) [14–16]. On the software side, there is an approach that uses a knowledge-based treatment plan with low variability [17, 18] and uses automatic planning [19] and a multicriteria optimization framework [20, 21] to reduce the frequency of planner intervention.

In this paper, we present an optimization method to handle not only dose-volume but also mean-dose constraints *directly* in IMRT treatment planning, which is an iterative algorithm derived from the discretization of a continuous-time dynamical system [22–29] with a set of equilibrium points. A theoretical proof for the convergence to an equilibrium corresponding to the desired IMRT planning is given by using the Lyapunov stability theorem. By introducing the concept of “*acceptable*,” which means the existence of a nonempty set of beam weights satisfying the given dose-volume and mean-dose constraints, and by using the proposed method for an acceptable IMRT planning, one can resolve the issue that the objective and evaluation are different in the conventional planning process. The system of nonlinear differential equations defined in this paper has a different vector field from that of the previously proposed system [29]. The previous method for obtaining an acceptable solution has a disadvantage in that it requires a long calculation time because of the high numerical cost of integrating piecewise differential equations describing the hybrid dynamical system. To resolve the disadvantage, we conduct a numerical discretization with multiplicative calculus [30, 31]. Moreover, for achieving a high-precision IMRT plan, we extend the previous continuous-time system to allow mean-dose as well as dose-volume concepts.

Now, we can get an acceptable solution for any totally acceptable IMRT treatment planning; however, we cannot obtain a nearly optimal solution close to the desired solution for every unacceptable planning. Therefore, as a strategy to search for such a solution, we present an achievement procedure. That is, when assuming that the target planning is totally unacceptable and partly acceptable except for one group of dose constraints, the objective is to get a solution located as close as possible to the remaining-one group unacceptable constraint while satisfying the partly acceptable situation. In considering the dynamics in the state space *Ω*, schematically shown in Figure 1, the first step of the procedure is to restrict the trajectory within the partly acceptable subspace *𝒜*_*e*_ using the proposed optimizing system for the objective function *U*_*e*_ such that the corresponding inverse problem is partly acceptable by excluding a function *U*_*r*_ from the total objective function with an acceptable set *𝒜*_*r*_ with *𝒜*_*e*_∩*𝒜*_*r*_ = *ϕ*. Then, the next step is to move the state *x* to decrease *U*_*r*_(*x*) and *U*_*e*_(*x*) in early and later iterations, respectively, by using the trajectory of an optimizing system, which has a time-dependent regularization effect [32] making it possible to optimize multiple criteria consisting of *U*_*e*_ and *U*_*r*_, with an initial value *a*_*e*_ in *𝒜*_*e*_. The optimizing system can get a desired solution in *𝒜*_*e*_ that is close to the optimal subspace *𝒜*_*r*_ for the remaining-one constraint function *U*_*r*_.

This paper is organized as follows. In Section 2, some preliminaries and definitions are provided. In Section 3, we propose a novel iterative method for obtaining an acceptable dose-volume and mean-dose constraint planning based on the continuous-time dynamical system, where the convergence to an acceptable set of solutions is theoretically guaranteed. A procedure is presented in Section 4 to get a nearly optimal solution for the remaining-one unacceptable constraint planning. In Sections 5 and 6, the performance of the proposed approach for an acceptable or unacceptable planning is confirmed through numerical experiments simulating a clinical setup. Finally, in Section 7, some concluding remarks are drawn.

In the rest of this section, we introduce notations that will be used below: (*θ*)_*k*_ indicates the *k*th element of the vector *θ*; and (Θ)_*i*_ and (Θ)^*j*^ indicate the *i*th row and *j*th column vectors of the matrix Θ, respectively.

## 2. IMRT Planning

The radiation oncologist performs IMRT planning to determine the PTV to be irradiated and the OARs to be spared. With IMRT, let *J* be the total number of beamlets that have split off from the radiation beam, and this is calculated as the number of delivered beams multiplied by the number of beamlets in each beam head. The problem of dose calculation, in matrix notation, has the form

(1) $$\begin{array}{c} D=Kx, \end{array}$$

where *D* ∈ *R*_+_^*I*^ with *R*_+_ being the set of nonnegative real numbers which is the dose vector whose components represent the total dose deposited in each voxel of the patient's three-dimensional volume, each component of $x\in \bar{\Omega }\subset R_{+}^{J}$ with $\bar{\Omega }$ indicating the closure of the open hypercube *Ω* = (0, *γ*)^*J*^ for some *γ* > 0 which represents the intensity in the corresponding beamlet, and *K* ∈ *R*_+_^*I*×*J*^ which consists of all elements *k*_*ij*_ representing the dose deposited in the *i*th voxel due to the unit intensity in the *j*th beamlet; it is called the dose influence (or deposition) matrix. If there are volumes of PTV and OAR with *I*_1_ and *I*_2_ voxels, respectively, then *D* includes *D*_1_ ∈ *R*_+_^*I*_1_^ and *D*_2_ ∈ *R*_+_^*I*_2_^ as subvectors, and *K* includes *K*_1_ ∈ *R*_+_^*I*_1_×*J*^ and *K*_2_ ∈ *R*_+_^*I*_2_×*J*^ as submatrices. A similar definition can be applied to the existence of multiple PTVs and OARs.

Let *b*_1_^*L*^ and *b*_2_^*U*^ represent the lower and upper bounds on the dose delivered to PTV and OAR, respectively (*b*_1_^*L*^ > 0 and *b*_2_^*U*^ ≥ 0). Additionally, we define an upper dose bound on the dose delivered to PTV as *b*_1_^*U*^ > *b*_1_^*L*^ to avoid excessively high doses inside the PTV. We also handle a mean dose denoted by ‖*D*_*m*_‖ as a real-valued function of the dose *D*_*m*_ ∈ *R*_+_^*I*_*m*_^, which is defined by

(2) $$\begin{array}{c} \left\|D_{m}\right\|≔\frac{1}{I_{m}}\overset{I_{m}}{\underset{i=1}{\sum }}\;{\left(D_{m}\right)}_{i}, \end{array}$$

for *m* = 1, 2. With respect to the mean-dose constraints, the lower and upper bounds on the mean dose of radiation delivered to PTV and OAR are indicated by *c*_1_^*L*^ and *c*_2_^*U*^, respectively.

**Definition 1 .**

The IMRT planning system {(*K*_1_, *b*_1_^*U*^), (*K*_1_, *b*_1_^*L*^), (*K*_2_, *b*_2_^*U*^), (*K*_1_, *c*_1_^*L*^), (*K*_2_, *c*_2_^*U*^)} is consistent if the set

(3) $$\begin{array}{c} E=\left\{e\in \Omega :\right.\;b_{1}^{U}\geq {\left(K_{1}\;e\right)}_{i_{1}}\geq b_{1}^{L},\;\forall i_{1}\in \left\{1,2,\cdots ,I_{1}\right\},\\ \;{\left(K_{2}\;e\right)}_{i_{2}}\leq b_{2}^{U},\;\forall i_{2}\in \left\{1,2,\cdots ,I_{2}\right\},\\ \;\left\|K_{1}e\right\|\geq c_{1}^{L},\\ \;\left.\left\|K_{2}e\right\|\leq c_{2}^{U}\right\} \end{array}$$

is not empty; otherwise, it is inconsistent.

**Definition 2 .**

For the given *x* ∈ *Ω* and each set of dose volumes and their conditions (*K*_1_, *b*_1_^*U*^, *ζ*_1_^*U*^), (*K*_1_, *b*_1_^*L*^, *ζ*_1_^*L*^), and (*K*_2_, *b*_2_^*U*^, *ζ*_2_^*U*^), where *ζ*_1_^*U*^ ≤ 1, *ζ*_1_^*L*^ ≤ 1, and *ζ*_2_^*U*^ ≤ 1 are the prescribed proportion rates, the corresponding dose distribution is partly dose-volume acceptable if each number of elements of the index sets

(4) $$\begin{array}{c} I_{1}^{U}\left(x\right)=\left\{i_{1}\in \left\{1,2,\cdots ,I_{1}\right\}\text{: }{\left(K_{1}\;x\right)}_{i_{1}}\leq b_{1}^{U}\right\},\\ I_{1}^{L}\left(x\right)=\left\{i_{1}\in \left\{1,2,\cdots ,I_{1}\right\}\text{: }{\left(K_{1}x\right)}_{i_{1}}\;\geq b_{1}^{L}\right\},\\ I_{2}^{U}\left(x\right)=\left\{i_{2}\in \left\{1,2,\cdots ,I_{2}\right\}\text{: }{\left(K_{2}\;x\right)}_{i_{2}}\leq b_{2}^{U}\right\} \end{array}$$

is, respectively, greater than the prescribed proportion of *I*_1_, *I*_1_, and *I*_2_, namely, each of the inequalities

(5) $$\begin{array}{c} \left|I_{1}^{U}\left(x\right)\right|\geq \zeta_{1}^{U}I_{1}, \end{array}$$

(6) $$\begin{array}{c} \left|I_{1}^{L}\left(x\right)\right|\geq \zeta_{1}^{L}I_{1},\; \end{array}$$

(7) $$\begin{array}{c} \left|I_{2}^{U}\left(x\right)\right|\geq \zeta_{2}^{U}I_{2} \end{array}$$

is satisfied for some *x*, where |·| indicates the number of elements in the set.

**Definition 3 .**

For the given *x* ∈ *Ω* and each set of doses and their conditions (*K*_1_, *c*_1_^*L*^) and (*K*_2_, *c*_2_^*U*^), the corresponding dose distribution is partly mean-dose acceptable if each of the inequalities

(8) $$\begin{array}{c} \left\|K_{1}\;x\right\|\geq c_{1}^{L},\\ \left\|K_{2}\;x\right\|\leq c_{2}^{U} \end{array}$$

is satisfied.

We define that the IMRT planning system is acceptable if there exists a common beam set such that the dose distributions in PTVs and OARs are partly dose-volume and mean-dose acceptable for all dose-volume and mean-dose constraints.

**Definition 4 .**

The IMRT planning system {(*K*_1_, *b*_1_^*U*^, *ζ*_1_^*U*^), (*K*_1_, *b*_1_^*L*^, *ζ*_1_^*L*^), (*K*_2_, *b*_2_^*U*^, *ζ*_2_^*U*^), (*K*_1_, *c*_1_^*L*^), (*K*_2_, *c*_2_^*U*^)} is acceptable if the following set is not empty:

(9) $$\begin{array}{c} A=\left\{a\in \Omega :\left|I_{1}^{U}\left(a\right)\right|\geq \zeta_{1}^{U}I_{1},\left|I_{1}^{L}\left(a\right)\right|\geq \zeta_{1}^{L}I_{1},\left|I_{2}^{U}\left(a\right)\right|\geq \zeta_{2}^{U}I_{2},\left\|K_{1}a\right\|\geq c_{1}^{L},\left\|K_{2}a\right\|\leq c_{2}^{U}\right\}. \end{array}$$

If the IMRT planning system is consistent, then it is acceptable. We are interested in the situation where the system is inconsistent and acceptable. In this paper, the problem of dose-volume and mean-dose constraint optimization in IMRT planning is defined to obtain the unknown variable *x* ∈ *𝒜* if the system is acceptable.

For describing the system, let us define the functions *P*_1_^*U*^(*D*_1_), *P*_1_^*L*^(*D*_1_), *P*_2_^*U*^(*D*_2_), *Q*_1_^*L*^(*D*_1_), and *Q*_2_^*U*^(*D*_2_) as follows:

(10) $$\begin{array}{c} {\left(P_{1}^{U}\left(D_{1}\right)\right)}_{i_{1}}=\left\{\begin{array}{cc} {\left(D_{1}\right)}_{i_{1}}, & \text{if }{\left(D_{1}\right)}_{i_{1}}\leq b_{1}^{U},\\ b_{1}^{U}, & \text{otherwise}, \end{array}\right.\\ {\left(P_{1}^{L}\left(D_{1}\right)\right)}_{i_{1}}=\left\{\begin{array}{cc} {\left(D_{1}\right)}_{i_{1}}, & \text{if }{\left(D_{1}\right)}_{i_{1}}\geq b_{1}^{L},\\ b_{1}^{L}, & \text{otherwise}, \end{array}\right.\\ {\left(P_{2}^{U}\left(D_{2}\right)\right)}_{i_{2}}=\left\{\begin{array}{cc} {\left(D_{2}\right)}_{i_{2}}, & \text{if }{\left(D_{2}\right)}_{i_{2}}\leq b_{2}^{U},\\ b_{2}^{U}, & \text{otherwise}, \end{array}\right.\\ {\left(Q_{1}^{L}\left(D_{1}\right)\right)}_{i_{1}}=\left\{\begin{array}{cc} {\left(D_{1}\right)}_{i_{1}}, & \text{if }\left\|D_{1}\right\|\geq c_{1}^{L},\\ \frac{c_{1}^{L}}{\left\|D_{1}\right\|}{\left(D_{1}\right)}_{i_{1}}, & \text{otherwise}, \end{array}\right.\\ {\left(Q_{2}^{U}\left(D_{2}\right)\right)}_{i_{2}}=\left\{\begin{array}{cc} {\left(D_{2}\right)}_{i_{2}}, & \text{if }\left\|D_{2}\right\|\leq c_{2}^{U},\\ \frac{c_{2}^{U}}{\left\|D_{2}\right\|}{\left(D_{2}\right)}_{i_{2}}, & \text{otherwise}, \end{array}\right. \end{array}$$

for *i*_1_ = 1, 2, ⋯, *I*_1_ and *i*_2_ = 1, 2, ⋯, *I*_2_. We consider the case where

(11) $$\begin{array}{c} D≔\left(\begin{array}{c} D_{1}\\ D_{1}\\ D_{2}\\ D_{1}\\ D_{2} \end{array}\right),\\ K≔\left(\begin{array}{c} K_{1}\\ K_{1}\\ K_{2}\\ K_{1}\\ K_{2} \end{array}\right), \end{array}$$

with *I* = 3*I*_1_ + 2*I*_2_. To simplify the description, we also define

(12) $$\begin{array}{c} P\left(D\right)≔\left(\begin{array}{c} P_{1}^{U}\left(D_{1}\right)\\ P_{1}^{L}\left(D_{1}\right)\\ P_{2}^{U}\left(D_{2}\right)\\ Q_{1}^{L}\left(D_{1}\right)\\ Q_{2}^{U}\left(D_{2}\right) \end{array}\right). \end{array}$$

## 3. IMRT Optimization for Acceptable Dose-Volume and Mean-Dose Constraint Planning

This section provides the definition of the dose-volume and mean-dose constraint optimization method and its theoretical results. Consider an initial-value problem for the nonlinear differential equation

(13) $$\begin{array}{c} \frac{dx_{j}\left(t\right)}{dt}=x_{j}\left(t\right)\left(1-\frac{x_{j}\left(t\right)}{\gamma }\right)\log\left(\frac{f_{j}\left(x\left(t\right)\right)}{\sigma_{j}}\right), \end{array}$$

where

(14) $$\begin{array}{c} f_{j}\left(x\right)=\overset{I_{1}}{\underset{i_{1}=1}{\sum }}\;{\left({\left(K_{1}\right)}^{j}\right)}_{i_{1}}{\left(\frac{{\left(P_{1}^{U}\left(K_{1}x\right)\right)}_{i_{1}}}{{\left(K_{1}x\right)}_{i_{1}}}\right)}^{R_{1}^{U}\left(x\right)}+\overset{I_{1}}{\underset{i_{1}=1}{\sum }}\;{\left({\left(K_{1}\right)}^{j}\right)}_{i_{1}}{\left(\frac{{\left(P_{1}^{L}\left(K_{1}x\right)\right)}_{i_{1}}}{{\left(K_{1}x\right)}_{i_{1}}}\right)}^{R_{1}^{L}\left(x\right)}+\overset{I_{2}}{\underset{i_{2}=1}{\sum }}\;{\left({\left(K_{2}\right)}^{j}\right)}_{i_{2}}{\left(\frac{{\left(P_{2}^{U}\left(K_{2}x\right)\right)}_{i_{2}}}{{\left(K_{2}x\right)}_{i_{2}}}\right)}^{R_{2}^{U}\left(x\right)}+\overset{I_{1}}{\underset{i_{1}=1}{\sum }}\;{\left({\left(K_{1}\right)}^{j}\right)}_{i_{1}}{\left(\frac{{\left(Q_{1}^{L}\left(K_{1}x\right)\right)}_{i_{1}}}{{\left(K_{1}x\right)}_{i_{1}}}\right)}^{S_{1}^{L}\left(x\right)}+\overset{I_{2}}{\underset{i_{2}=1}{\sum }}\;{\left({\left(K_{2}\right)}^{j}\right)}_{i_{2}}{\left(\frac{{\left(Q_{2}^{U}\left(K_{2}x\right)\right)}_{i_{2}}}{{\left(K_{2}x\right)}_{i_{2}}}\right)}^{S_{2}^{U}\left(x\right)},\\ \sigma_{j}=3\overset{I_{1}}{\underset{i_{1}=1}{\sum }}\;{\left({\left(K_{1}\right)}^{j}\right)}_{i_{1}}+2\overset{I_{2}}{\underset{i_{2}=1}{\sum }}\;{\left({\left(K_{2}\right)}^{j}\right)}_{i_{2}}, \end{array}$$

for *j* = 1, 2, ⋯, *J* with *x*(0) = *x*^0^ ∈ *Ω*. Where

(15) $$\begin{array}{c} R_{1}^{U}\left(x\right)=\left\{\begin{array}{cc} 0, & \text{if }x\text{ with }\left(K_{1},b_{1}^{U},\zeta_{1}^{U}\right)\text{ is partly dose}‐\text{volume acceptable},\\ 1, & \text{otherwise}, \end{array}\right.\\ R_{1}^{L}\left(x\right)=\left\{\begin{array}{cc} 0, & \text{if }x\text{ with }\left(K_{1},b_{1}^{L},\zeta_{1}^{L}\right)\text{ is partly dose}‐\text{volume acceptable},\\ 1, & \text{otherwise}, \end{array}\right.\\ R_{2}^{U}\left(x\right)=\left\{\begin{array}{cc} 0, & \text{if }x\text{ with }\left(K_{2},b_{2}^{U},\zeta_{2}^{U}\right)\text{ is partly dose}‐\text{volume acceptable},\\ 1, & \text{ otherwise}, \end{array}\right.\\ S_{1}^{L}\left(x\right)=\left\{\begin{array}{cc} 0, & \text{if }x\text{ with }\left(K_{1},c_{1}^{L}\right)\text{ is partly mean}‐\text{dose acceptable},\\ 1, & \text{otherwise}, \end{array}\right.\\ S_{2}^{U}\left(x\right)=\left\{\begin{array}{cc} 0, & \text{if }x\text{ with }\left(K_{2},c_{2}^{U}\right)\text{ is partly mean}‐\text{dose acceptable},\\ 1, & \text{otherwise}, \end{array}\right. \end{array}$$

for *i*_1_ = 1, 2, ⋯, *I*_1_ and *i*_2_ = 1, 2, ⋯, *I*_2_.

We give theoretical results for the behavior of the solution to the dynamical system in Equation (13). First, we show that all solutions stay inside the hypercube.

**Proposition 1 .**

If we choose the initial value *x*^0^ ∈ *Ω* of the dynamical system in Equation (13), then the solution *φ*(*t*, *x*^0^) stays in *Ω* for all *t* > 0.

**Proof**

Since the system can be written as *dx*_*j*_/*dt* = *x*_*j*_(1 − *γ*^−1^*x*_*j*_)*h*_*j*_(*x*) with a function *h*_*j*_, we see that for any *j*, the solution satisfies *dφ*_*j*_/*dt* ≡ 0 on the subspace where *x*_*j*_ = 0 or *x*_*j*_ = *γ*. Therefore, the subspace is invariant, and trajectories cannot pass through every invariant subspace in accordance with the uniqueness of solutions for the initial-value problem. This leads to any solution *φ*(*t*, *x*^0^) of the system in Equation (13) with initial value *x*^0^ ∈ *Ω* being in *Ω* for all *t* > 0.

Next, we prove the stability of equilibrium in the set *𝒜*, which corresponds to the desired radiation beam weights. Namely, the existence of a Lyapunov function for the system in Equation (13) guarantees the stability of the equilibrium set [33].

**Theorem 1 .**

If the IMRT planning system is acceptable, then *𝒜* in Equation (9) as an equilibrium set of Equation (13) is stable.

**Proof**

Any point *a* ∈ *𝒜* is an equilibrium of Equation (13), so we can say that *𝒜* is an equilibrium set of equilibrium points. Consider a Lyapunov-candidate function defined in the set *Ω* as

(16) $$\begin{array}{c} V\left(x\right)=\overset{J}{\underset{j=1}{\sum }}\;\sigma_{j}\left(a_{j}\log\frac{a_{j}}{x_{j}}+\left(\gamma -a_{j}\right)\log\frac{\gamma -a_{j}}{\gamma -x_{j}}\right)=\overset{J}{\underset{j=1}{\sum }}\;\sigma_{j}\int_{a_{j}}^{x_{j}}\;\left(\frac{v-a_{j}}{v}+\frac{v-a_{j}}{\gamma -v}\right)dv=\overset{J}{\underset{j=1}{\sum }}\;\sigma_{j}\int_{a_{j}}^{x_{j}}\;\frac{\gamma \left(v-a_{j}\right)}{v\left(\gamma -v\right)}dv, \end{array}$$

which is positive definite with respect to the point *a* ∈ *𝒜*. We obtain its derivative along the solution to the system in Equation (13). When *x* ∈ *Ω* is neither partly dose-volume nor mean-dose acceptable, the derivative is given by

(17) $$\begin{array}{c} {\left.\dot{V}\left(x\right)\right|}_{\left(13\right)}=\overset{J}{\underset{j=1}{\sum }}\;\sigma_{j}\frac{\gamma \left(x_{j}-a_{j}\right)}{x_{j}\left(\gamma -x_{j}\right)}{\dot{x}}_{j}=-\overset{J}{\underset{j=1}{\sum }}\;a_{j}\sigma_{j}\log\left(\sigma_{j}^{-1}\overset{I}{\underset{i=1}{\sum }}\;{\left({\left(K\right)}^{j}\right)}_{i}\frac{{\left(P\left(Kx\right)\right)}_{i}}{{\left(Kx\right)}_{i}}\right)+\overset{J}{\underset{j=1}{\sum }}\;x_{j}\sigma_{j}\log\left(\sigma_{j}^{-1}\overset{I}{\underset{i=1}{\sum }}\;{\left({\left(K\right)}^{j}\right)}_{i}\frac{{\left(P\left(Kx\right)\right)}_{i}}{{\left(Kx\right)}_{i}}\right)\leq -\overset{J}{\underset{j=1}{\sum }}\;a_{j}\sigma_{j}\left(\sigma_{j}^{-1}\overset{I}{\underset{i=1}{\sum }}\;{\left({\left(K\right)}^{j}\right)}_{i}\left(\log\left({\left(P\left(Kx\right)\right)}_{i}\right)-\log\left({\left(Kx\right)}_{i}\right)\right)\right)+\overset{J}{\underset{j=1}{\sum }}\;x_{j}\sigma_{j}\left(\sigma_{j}^{-1}\left(\overset{I}{\underset{i=1}{\sum }}\;{\left(\left(K^{j}\right)\right)}_{i}\frac{{\left(P\left(Kx\right)\right)}_{i}}{{\left(Kx\right)}_{i}}\right)-1\right)\leq -\overset{I}{\underset{i=1}{\sum }}\;{\left(Ka\right)}_{i}\left(\log\left({\left(P\left(Kx\right)\right)}_{i}\right)-\log\left({\left(Kx\right)}_{i}\right)\right)+\overset{I}{\underset{i=1}{\sum }}\;{\left(Kx\right)}_{i}\left(\frac{{\left(P\left(Kx\right)\right)}_{i}}{{\left(Kx\right)}_{i}}-1\right)\leq -\overset{I}{\underset{i=1}{\sum }}\;{\left(Ka\right)}_{i}\left(1-\frac{{\left(Kx\right)}_{i}}{{\left(P\left(Kx\right)\right)}_{i}}\right)+\overset{I}{\underset{i=1}{\sum }}\;{\left(Kx\right)}_{i}\left(\frac{{\left(P\left(Kx\right)\right)}_{i}}{{\left(Kx\right)}_{i}}-1\right)=-\overset{I}{\underset{i=1}{\sum }}\;\frac{1}{{\left(P\left(Kx\right)\right)}_{i}}\left({\left(Kx\right)}_{i}-{\left(P\left(Kx\right)\right)}_{i}\right)\left({\left(P\left(Kx\right)\right)}_{i}-{\left(Ka\right)}_{i}\right). \end{array}$$

To treat any *x* ∈ *Ω*, define the index sets:

(18) $$\begin{array}{c} {\bar{I}}_{1}^{U}\left(x\right)=\left\{\begin{array}{cc} \phi , & \text{if }x\text{ with }\left(K_{1},b_{1}^{U},\zeta_{1}^{U}\right)\text{ is partly dose}‐\text{volume acceptable},\\ \left\{1,2,\cdots ,I_{1}\right\}\backslash I_{1}^{U}\left(x\right), & \text{otherwise}, \end{array}\right.\\ {\bar{I}}_{1}^{L}\left(x\right)=\left\{\begin{array}{cc} \phi , & \text{if }x\text{ with }\left(K_{1},b_{1}^{L},\zeta_{1}^{L}\right)\text{ is partly dose}‐\text{volume acceptable},\\ \left\{1,2,\cdots ,I_{1}\right\}\backslash I_{1}^{L}\left(x\right), & \text{otherwise}, \end{array}\right.\\ {\bar{I}}_{2}^{U}\left(x\right)=\left\{\begin{array}{cc} \phi , & \text{if }x\text{ with }\left(K_{2},b_{2}^{U},\zeta_{2}^{U}\right)\text{ is partly dose}‐\text{volume acceptable},\\ \left\{1,2,\cdots ,I_{2}\right\}\backslash I_{2}^{U}\left(x\right), & \text{otherwise}, \end{array}\right.\\ {\overset{¯}{O}}_{1}^{L}\left(x\right)=\left\{\begin{array}{cc} \phi , & \text{if }x\text{ with }\left(K_{1},c_{1}^{L}\right)\text{ is partly mean}‐\text{dose acceptable},\\ \left\{1,2,\cdots ,I_{1}\right\}, & \text{otherwise}, \end{array}\right.\\ {\overset{¯}{O}}_{2}^{U}\left(x\right)=\left\{\begin{array}{cc} \phi , & \text{if }x\text{ with }\left(K_{2},c_{2}^{U}\right)\text{ is partly mean}‐\text{dose acceptable},\\ \left\{1,2,\cdots ,I_{2}\right\}, & \text{otherwise}. \end{array}\right. \end{array}$$

Then, the calculation of the derivative is reduced to the following:

(19) $$\begin{array}{c} {\left.\dot{V}\left(x\right)\right|}_{\left(13\right)}=-\frac{1}{b_{1}^{U}}\underset{i_{1}\in {\bar{I}}_{1}^{U}\left(x\right)}{\sum }\;\left({\left(K_{1}x\right)}_{i_{1}}-b_{1}^{U}\right)\left(b_{1}^{U}-{\left(K_{1}a\right)}_{i_{1}}\right)-\frac{1}{b_{1}^{L}}\underset{i_{1}\in {\bar{I}}_{1}^{L}\left(x\right)}{\sum }\;\left(b_{1}^{L}-{\left(K_{1}x\right)}_{i_{1}}\right)\left({\left(K_{1}a\right)}_{i_{1}}-b_{1}^{L}\right)-\frac{1}{b_{2}^{U}}\underset{i_{2}\in {\bar{I}}_{2}^{U}\left(x\right)}{\sum }\;\left({\left(K_{2}x\right)}_{i_{2}}-b_{2}^{U}\right)\left(b_{2}^{U}-{\left(K_{2}a\right)}_{i_{2}}\right)-\frac{1}{c_{1}^{L}}\left(c_{1}^{L}-\left\|K_{1}x\right\|\right)\underset{i_{1}\in {\overset{¯}{O}}_{1}^{L}\left(x\right)}{\sum }\;{\left(K_{1}a\right)}_{i_{1}}-\frac{c_{1}^{L}}{\left\|K_{1}x\right\|}{\left(K_{1}x\right)}_{i_{1}}-\frac{1}{c_{2}^{U}}\left(\left\|K_{2}x\right\|-c_{2}^{U}\right)\underset{i_{2}\in {\overset{¯}{O}}_{2}^{U}\left(x\right)}{\sum }\;\frac{c_{2}^{U}}{\left\|K_{2}x\right\|}{\left(K_{2}x\right)}_{i_{2}}-{\left(K_{2}a\right)}_{i_{2}}\leq 0. \end{array}$$

The last inequality is supported by

(20) $$\begin{array}{c} \overset{I_{1}}{\underset{i_{1}=1}{\sum }}\;{\left(K_{1}a\right)}_{i_{1}}-\frac{c_{1}^{L}}{\left\|K_{1}x\right\|}{\left(K_{1}x\right)}_{i_{1}}=I_{1}\left(\left\|K_{1}a\right\|-c_{1}^{L}\right)>0,\\ \overset{I_{2}}{\underset{i_{2}=1}{\sum }}\;\frac{c_{2}^{U}}{\left\|K_{2}\;x\right\|}{\left(K_{2}x\right)}_{i_{2}}-{\left(K_{2}a\right)}_{i_{2}}=I_{2}\left(c_{2}^{U}-\left\|K_{2}a\right\|\right)>0, \end{array}$$

for partly mean-dose unacceptable (*K*_1_, *c*_1_^*L*^) and (*K*_2_, *c*_2_^*U*^). The derivative is zero at *x* = *a* ∈ *Ω*. Thus, *V*(*x*) is a Lyapunov function with respect to *a*. Consequently, the equilibrium set *𝒜* is stable.

A numerical discretization of differential equations describing the system in Equation (13) derives an iterative method. By using geometric multiplicative Euler discretization [30, 31], we obtain the iterative algorithm of the variable *z* ∈ *Ω* for radiation beam weight

(21) $$\begin{array}{c} z_{j}\left(n+1\right)=z_{j}\left(n\right)\exp{\left(\left(1-\frac{z_{j}\left(n\right)}{\gamma }\right)\log\left(\frac{f_{j}\left(z\left(n\right)\right)}{\sigma_{j}}\right)\right)}^{h}, \end{array}$$

for *j* = 1, 2, ⋯, *J* and *n* = 0, 1, 2, ⋯ with *z*(0) = *x*^0^ ∈ *Ω*, where *h* > 0 denotes a step size. When *γ*⟶∞, *h* = 1, and all binary functions *R*_1_^*U*^, *R*_1_^*L*^, *R*_1_^*U*^, *S*_1_, and *S*_2_^*U*^ are assumed to be one for simplicity, the *j*th element of *z* can be described as

(22) $$\begin{array}{c} z_{j}\left(n+1\right)=\frac{z_{j}\left(n\right)}{\sum_{i=1}^{I}\;{\left({\left(K\right)}^{j}\right)}_{i}}\overset{I}{\underset{i=1}{\sum }}\;{\left({\left(K\right)}^{j}\right)}_{i}\frac{{\left(P\left(Kz\left(n\right)\right)\right)}_{i}}{{\left(Kz\left(n\right)\right)}_{i}}, \end{array}$$

for *j* = 1, 2, ⋯, *J*. We see that the iterative formula in Equation (22) is similar to that of the expectation-maximization (EM) method in computed tomography. Namely, replacing *P*(*Kz*(*n*)) with the measured projection and assuming *K* and *z* are the projection operator and pixel density of the image to be reconstructed, respectively, the iterative formula describes the EM-type reconstruction algorithm.

One can design a different combination of vector field and Lyapunov function from that of Equations (13) and (16). For example, a continuous analog of the iterative gradient algorithm based on the split feasibility problem [11] for handling dose constraints is able to be a continuous-time system with an equilibrium whose stability is supported by the Lyapunov theorem, but it is required to choose an appropriate value of the step size in the iterative formula as an additive Euler discretization for avoiding slow convergence and oscillatory behavior in solutions. Our resultant iterative algorithm as a modification of the EM procedure, which is a popular iterative image reconstruction method in practice, is expected to calculate the desired solution with a good convergence rate [34], when *h* = 1.

## 4. IMRT Optimization for Remaining-One Unacceptable Dose-Volume and Mean-Dose Constraint Planning

Consider an IMRT planning system

(23) $$\begin{array}{c} S≔\left\{\left(K_{1},b_{1}^{U},\zeta_{1}^{U}\right),\left(K_{1},b_{1}^{L},\zeta_{1}^{L}\right),\left(K_{2},b_{2}^{U},\zeta_{2}^{U}\right),\left(K_{1},c_{1}^{L}\right),\left(K_{2},c_{2}^{U}\right),\left(K_{3},b_{3}^{U},\zeta_{3}^{U}\right),\left(K_{3},c_{3}^{U}\right)\right\}, \end{array}$$

where the subsystem

(24) $$\begin{array}{c} \left\{\left(K_{3},b_{3}^{U},\zeta_{3}^{U}\right),\left(K_{3},c_{3}^{U}\right)\right\}≕S_{r}, \end{array}$$

indicates an additional set of dose-volume and mean-dose constraints with the upper bound for an OAR, as an example of remaining-one unacceptable constraint, by rearranging the formulation described in Section 3. We assume that the planning system is totally unacceptable and the subsystem

(25) $$\begin{array}{c} S_{e}≔S\backslash S_{r}=\left\{\left(K_{1},b_{1}^{U},\zeta_{1}^{U}\right),\left(K_{1},b_{1}^{L},\zeta_{1}^{L}\right),\left(K_{2},b_{2}^{U},\zeta_{2}^{U}\right),\left(K_{1},c_{1}^{L}\right),\left(K_{2},c_{2}^{U}\right)\right\}, \end{array}$$

is acceptable. We show a procedure to get a solution located as close as possible to the remaining-one unacceptable constraint of *S*_*r*_ while satisfying the partly acceptable situation as in the subsystem *S*_*e*_. In the procedure, we use an initial value problem for the following difference equation of variables *z*(*n*) with initial state *z*(*N*_1_) ∈ *Ω* starting at *N*_1_ ≥ 0:

(26) $$\begin{array}{c} z_{j}\left(n+1\right)=z_{j}\left(n\right)\exp{\left(\left(1-\frac{z_{j}\left(n\right)}{\gamma }\right)\log\left(\frac{f_{j}\left(z\left(n\right)\right)+g_{j}\left(z\left(n\right)\right)}{\sigma_{j}+\delta_{j}}\right)\right)}^{h}, \end{array}$$

for *n* = *N*_1_, *N*_1_ + 1, ⋯, where the functions *g*_*j*_ and *δ*_*j*_ are, respectively, defined by

(27) $$\begin{array}{c} g_{j}\left(z\right)=\overset{I_{3}}{\underset{i_{3}=1}{\sum }}\;{\left({\left(K_{3}\right)}^{j}\right)}_{i_{3}}{\left(\frac{{\left(P_{3}^{U}\left(K_{3}z\right)\right)}_{i_{3}}}{{\left(K_{3}z\right)}_{i_{3}}}\right)}^{R_{3}^{U}\left(z\right)}+\overset{I_{3}}{\underset{i_{3}=1}{\sum }}\;{\left({\left(K_{3}\right)}^{j}\right)}_{i_{3}}{\left(\frac{{\left(Q_{3}^{U}\left(K_{3}z\right)\right)}_{i_{3}}}{{\left(K_{3}z\right)}_{i_{3}}}\right)}^{S_{3}^{U}\left(z\right)},\\ \delta_{j}=2\overset{I_{3}}{\underset{i_{3}=1}{\sum }}\;{\left({\left(K_{3}\right)}^{j}\right)}_{i_{3}}, \end{array}$$

for *j* = 1, 2, ⋯, *J*. Where

(28) $$\begin{array}{c} {\left(P_{3}^{U}\left(D_{3}\right)\right)}_{i_{3}}=\left\{\begin{array}{cc} {\left(D_{3}\right)}_{i_{3}}, & \text{if }{\left(D_{3}\right)}_{i_{3}}\leq b_{3}^{U},\\ b_{3}^{U}, & \text{otherwise}, \end{array}\right.\\ {\left(Q_{3}^{U}\left(D_{3}\right)\right)}_{i_{3}}=\left\{\begin{array}{cc} {\left(D_{3}\right)}_{i_{3}}, & \text{if }\left\|D_{3}\right\|\leq c_{3}^{U},\\ \frac{c_{3}^{U}}{\left\|D_{3}\right\|}{\left(D_{3}\right)}_{i_{3}}, & \text{otherwise}, \end{array}\right. \end{array}$$

for *i*_3_ = 1, 2, ⋯, *I*_3_ and

(29) $$\begin{array}{c} R_{3}^{U}\left(z\left(n\right)\right)=\left\{\begin{array}{cc} 0, & \text{if }z\text{ with }\left(K_{3},b_{3}^{U},\zeta_{3}^{U}\right)\text{ is partly dose}‐\text{volume acceptable},\\ \lambda^{n-N_{1}}, & \text{otherwise}, \end{array}\right.\\ S_{3}^{U}\left(z\left(n\right)\right)=\left\{\begin{array}{cc} 0, & \text{if }z\text{ with }\left(K_{3},c_{3}^{U}\right)\text{ is partly mean}‐\text{dose acceptable},\\ \lambda^{n-N_{1}}, & \text{otherwise}, \end{array}\right. \end{array}$$

with a positive parameter *λ*. Note that one takes *λ*^*n*^⟶0 and then has *g*_*j*_(*z*(*n*))⟶*δ*_*j*_, *j* = 1, 2, ⋯, *J*, for *n*⟶∞, when *λ* < 1. We give the procedure as follows:

**Procedure 1 .**

For an IMRT planning system *S* consisting of Equation (23), which is totally unacceptable and has a partly acceptable subsystem *S*_*e*_ in Equation (25), the following shows a procedure for obtaining a solution located as close as possible to the remaining-one unacceptable constraint of *S*_*r*_ in Equation (24) while satisfying the partly acceptable situation as in the subsystem *S*_*e*_.

**Step 1 .**

The first step of the procedure is to solve iterative solutions to the difference equation in Equation (21) for the subsystem *S*_*e*_ and obtain a stable fixed point *a*_*e*_ in the set *𝒜*_*e*_ illustrated in Figure 1. Obtaining *a*_*e*_ ∈ *𝒜*_*e*_ is guaranteed by Theorem 6 for the continuous analog of the difference system in Equation (21).

**Step 2 .**

The next step is to examine the iterative algorithm in Equation (26) with some value of the parameter *λ* < 1 and an initial value *z*(*N*_1_) = *a*_*e*_ ∈ *𝒜*_*e*_ and move the state *z*(*N*_1_ + *n*), *n* = 1, 2, ⋯, *N*_2_, while expecting the decrease of the objective function *U*_*r*_(*z*(*N*_1_ + *n*)), as shown in Figure 1. Note that because the partly acceptable situation of the subsystem *S*_*e*_ means that *f*_*j*_(*z*) = *σ*_*j*_ in Equation (26) at *z* = *a*_*e*_ ∈ *𝒜*_*e*_ for *j* = 1, 2, ⋯, *J*, the iterative steps can forcibly decrease the sequence {*U*_*r*_(*z*(*n*))}_*n*=*N*_1__^*N*_1_+*ν*^ for at least a small value of *ν*. By introducing the function *g*_*j*_(*z*(*n*)) with a time-varying parameter *λ*^*n*−*N*_1_^ in Equation (26), the iterative process has a time-dependent regularization effect making it possible to optimize multiple criteria. As the function tends to *δ*_*j*_ independently of *z*(*n*) along with time *n* that has passed, the optimizing system can get a desired solution in *𝒜*_*e*_ that is close to the optimal subspace *𝒜*_*r*_ with respect to the objective function *U*_*r*_ for the remaining-one constraint.

## 5. Experimental Method

To evaluate the proposed method, we examine two IMRT treatment planning problems: “acceptable planning” and “remaining-one unacceptable planning.” Figure 2 shows 128 × 128-sized phantom images for the planning study. The image in Figure 2(a) shows a phantom consisting of a core (blue region) and C-shape PTV (red region), which refers to a C-shape phantom published in the task group 119 report [35] from the American Association of Physicists in Medicine (AAPM). The image in Figure 2(b) represents a phantom simulating a head and neck with a PTV, parotid gland, and spinal cord, which are colored red, green, and blue, respectively. The former image was used for an acceptable planning, and the latter was used for a partly unacceptable planning. In many clinical cases, an ideal solution to an IMRT planning problem is not achieved; therefore, planning for IMRT requires a trial-and-error process to find a solution for “partly acceptable planning.” Generally, it is necessary for a planner to set priorities for each of the PTVs and OARs. For example, in the case of a simple structure phantom, such as the C-shape phantom, an ideal and feasible solution is obtained (“acceptable planning”) because the PTV and core can be handled with equal priority. However, in the case of a complex structure phantom, such as the head and neck phantoms, there is a case where the DVCs of other organs cannot be satisfied by achieving the DVCs of a high-priority organ. In this case, a planner prioritizes the PTV and spinal cord, and the parotid's DVC is set to the next. In other words, the IMRT planning that satisfies the DVCs of the PTV and cord perfectly achieves the parotid's DVC as much as possible. This is valuable because if the spinal cord is irradiated excessively, the risk of myelopathy caused by radiation will increase. In addition, to reduce the dose applied to the parotid gland as much as possible, the function of the salivary glands can be preserved [36–42].

Table 1 shows the DVCs for the C-shape phantom case, and we adopted a 9-field beam arrangement with every 40-degree beam from 0 to 360 degrees, which is given as a harder version of the problem in the task group 119 report [35].  Table 2 shows the DVCs and mean doses for the head and neck phantom case. To achieve more stringent DVCs, we adopted a 36-field beam arrangement with every 5-degree beam from 0 to 175 degrees. Although there is research related to beam angle optimization in IMRT [43], the objective of the beam arrangement is to obtain dose distributions equivalent or superior to static gantry IMRT [3–5]. So we adopted a VMAT technique to perform complex treatment planning.

## 6. Experimental Results and Discussion

We used the iterative solutions *z*(*n*), *n* = 0, 1, 2, ⋯, to the algorithms described by Equations (21) and (26) with *h* = 1 and *z*(0) = *x*^0^ for solving the IMRT inverse problems of acceptable and remaining-one unacceptable plannings, respectively. The initial values of *x*^0^ were commonly chosen as *x*_*j*_^0^ = 0.1 for any *j*, unless otherwise specified.

### 6.1. Acceptable Planning

We first examined solving the problem of acceptable IMRT planning using the harder condition defined by AAPM, as shown in Table 1, with the C-shape phantom in Figure 2(a). The AAPM report [35] says that “the goal of this problem set is probably not achievable and tests a system that is being pushed very hard,” but it is acceptable in the meaning of Definition 4. Actually, we obtained the dose-volume histograms (DVHs) showing that the dose distributions of PTV and OAR (core) perfectly satisfy all prescribed DVCs (see Figure 3) generated by using the solution *z*(500).  Figure 4 shows the iterative evolution of the divergence *V*(*z*) defined in Equation (16), which is a Lyapunov function of the continuous analog described in Equation (13). The monotonic decrease of the divergence with solutions toward a fixed point in the set *𝒜* confirms the theoretical result of Theorem 6 and guarantees an appropriate discretization of the differential equation.

The evolutions of the dose-volume proportion rates

(30) $$\begin{array}{c} \frac{\left|I_{1}^{U}\left(z\left(n\right)\right)\right|}{I_{1}},\frac{\left|I_{1}^{L}\left(z\left(n\right)\right)\right|}{I_{1}},\frac{\left|I_{2}^{U}\left(z\left(n\right)\right)\right|}{I_{2}},\;n=0,1,2,\cdots ,500, \end{array}$$

for DVCs with (*K*_1_, *b*_1_^*U*^, *ζ*_1_^*U*^), (*K*_1_, *b*_1_^*L*^, *ζ*_1_^*L*^), and (*K*_2_, *b*_2_^*U*^, *ζ*_2_^*U*^) are, respectively, shown in the upper panel of Figure 5. We see that each proportion rate behaves to become greater than the prescribed rate (red line in the graph) as the number of iteration steps increases. The dose distribution satisfying Equation (5) implies a partly dose-volume acceptability according to Definition 2 and is confirmed by each graph of binary functions *R*_1_^*U*^(*z*(*n*)), *R*_1_^*L*^(*z*(*n*)), and *R*_2_^*U*^(*z*(*n*)) as shown in the lower panel of Figure 5. When all dose distributions become partly dose-volume acceptable, then every binary function is exactly zero after the iterative solution has reached a fixed point in *𝒜*.

### 6.2. Remaining-One Unacceptable Planning

The proposed Procedure 7 in Section 4 was experimentally demonstrated by applying it to a remaining-one unacceptable dose-volume and mean-dose constraint planning for the head and neck phantoms in Figure 2(b) with constraints given in Table 2.

Figure 6 shows DVHs obtained from a solution *z*(1000) to the algorithm in Equation (26) with *λ* = 1, *N*_1_ = 0, and *z*(0) = *x*^0^ for the totally unacceptable planning *S* defined in Equation (23). The resultant values *V*_75_ = 28% and *V*_70_ = 67% at PTV, *V*_30_ = 1% at OAR (spinal cord), and so on are not satisfied with the prescribed constraints except for *D*_mean_ = 5.7 Gy at OAR (parotid). Because the achievement of constraints for PTV and OAR (spinal cord) are mandatory based on the overall objective, we tried to examine an inverse problem for optimizing the subsystem *S*_*e*_ in Equation (25) using a fixed point *z*(100) ∈ *𝒜*_*e*_ applied to the algorithm described in Equation (21). As shown in Figure 7 (which indicates DVHs), the dose distributions of PTV and OAR (spinal cord) fulfill the prescribed conditions as expected; however, the results of *V*_5_ = 100% and *D*_mean_ = 50 Gy at OAR (parotid) are clinically unsatisfactory. For the perfect satisfaction of dose-volume and mean-dose constraints at PTV and OAR (spinal cord) being kept while the dose distribution at OAR (parotid) is reduced without causing the user's trial and error, we performed an experiment according to the proposed procedure. The value of the parameter *λ* in Equation (21) used in Step 2 of Procedure 7 was set to 0.9, unless otherwise noted. The solution *z*(1000) obtained after the procedure was used for calculating DVHs, as shown in Figure 8. We see that the dose distributed to OAR (parotid) was less than that shown in Figure 7(c). Actually, *D*_mean_ at OAR (parotid) can be decreased to 29 Gy from 50 Gy owing to the procedure. It is reported that a lower mean dose of the parotid gland is more effective for avoiding mouth dryness caused by salivary gland disorder [42]. Moreover, one can prevent a salivary disorder by reducing the mean doses to be applied to the parotid gland so that they are as small as possible [37, 38].

For evaluating the effectiveness of the proposed procedure quantitatively, we drew the graph in Figure 9 showing the evolution of the distances

(31) $$\begin{array}{c} U_{e}\left(z\right)=R_{1}^{U}\left(z\right)\overset{I_{1}}{\underset{i_{1}=1}{\sum }}\;{\left({\left(P_{1}^{U}\left(K_{1}z\right)\right)}_{i_{1}}-{\left(K_{1}z\right)}_{i_{1}}\right)}^{2}+R_{1}^{L}\left(z\right)\overset{I_{1}}{\underset{i_{1}=1}{\sum }}\;{\left({\left(P_{1}^{L}\left(K_{1}z\right)\right)}_{i_{1}}-{\left(K_{1}z\right)}_{i_{1}}\right)}^{2}+R_{2}^{U}\left(z\right)\overset{I_{2}}{\underset{i_{2}=1}{\sum }}\;{\left({\left(P_{2}^{U}\left(K_{2}z\right)\right)}_{i_{2}}-{\left(K_{2}z\right)}_{i_{2}}\right)}^{2}+S_{2}^{U}\left(z\right)\overset{I_{2}}{\underset{i_{2}=1}{\sum }}\;{\left({\left(Q_{2}^{U}\left(K_{2}z\right)\right)}_{i_{2}}-{\left(K_{2}z\right)}_{i_{2}}\right)}^{2},\\ U_{r}\left(z\right)=R_{3}^{U}\left(z\right)\overset{I_{3}}{\underset{i_{3}=1}{\sum }}\;{\left({\left(P_{3}^{U}\left(K_{3}z\right)\right)}_{i_{3}}-{\left(K_{3}z\right)}_{i_{3}}\right)}^{2}+S_{3}^{U}\left(z\right)\overset{I_{3}}{\underset{i_{3}=1}{\sum }}\;{\left({\left(Q_{3}^{U}\left(K_{3}z\right)\right)}_{i_{3}}-{\left(K_{3}z\right)}_{i_{3}}\right)}^{2}, \end{array}$$

each of which is defined as a squared *L*_2_ norm. The values of *U*_*e*_(*z*) and *U*_*r*_(*z*) become zero if and only if the solutions *z* to the subsystems *S*_*e*_ and *S*_*r*_ are in the acceptable sets *𝒜*_*e*_ and *𝒜*_*r*_, respectively. In the figure, the numbers of iteration *n* in the ranges [0, *N*_1_] and [*N*_1_, 1000] where *N*_1_ = 100 are, respectively, in Steps 1 and 2 of Procedure 7. We see that the iterative sequence {*z*(*n*)}_*n*=0_^*N*_1_^ converges to the subspace *𝒜*_*e*_ with decreasing {*U*_*e*_(*z*(*n*))}_*n*=0_^*N*_1_^ by applying the process of Step 1 for obtaining an initial state of Step 2. In Step 2, {*U*_*r*_(*z*(*n*))}_*n*=*N*_1__^*N*_1_+27^ is drastically decreased although the solution overflows from *𝒜*_*e*_, and {*U*_*e*_(*z*(*n*))}_*n*=*N*_1__^*N*_1_+5^ is slightly increased. The remaining iterations are for making the solution converge to *𝒜*_*e*_ again. Note that the maximum of the sequence {*U*_*r*_(*z*(*n*))}_*n*=*N*_1_+27_^1000^ results in a small value compared to the decrease caused in the preceding iterations.

We show how selecting the parameter value affects the performance with respect to decreasing the cost function.  Figure 10 illustrates the relation between *λ* and *U*_*r*_(*z*(*N*_1_ + *N*_2_)) where *N*_2_ denotes the iteration number at which the solution to Equation (26) with initial state *z*(*N*_1_) has fallen into the partly acceptable set *𝒜*_*e*_. From the figure, we observe that a larger *λ* leads to a smaller value of the resultant *U*_*r*_, while being accompanied with a larger number of iterations, *N*_2_, for the convergence.

## 7. Conclusion

For handling dose-volume and mean-dose constraints directly in the optimization of IMRT treatment inverse planning, we have proposed a novel iterative algorithm derived from the discretization of a continuous-time dynamical system. The proposed system has an advantage in that the stability of an equilibrium corresponding to the desired optimal solution to the inverse problem is able to be proven using the Lyapunov theorem. Through numerical experiments with the C-shape phantom (AAPM TG-119) for an acceptable planning and an extended C-shape phantom simulating the head and neck for remaining-one unacceptable planning, we confirmed that we can obtain an optimal solution and a nearly optimal solution located as close as possible to the remaining-one unacceptable constraint.

Our approach presented in this paper enables us to develop an iterative method of IMRT optimization by discretizing a continuous-time system in which the global stability of a desired equilibrium is guaranteed based on the dynamical system theory. The advantage of the approach is due to the Lyapunov theorem that establishes the stability of equilibrium if there exists a Lyapunov function even for a hybrid dynamical system. The direct construction of iterative algorithms with a theoretical guarantee of convergence for a given objective function including inequalities with percentages is generally difficult. Although a drawback of the dynamical system approach is that finding a combination of a vector field and Lyapunov function is generally a hard problem, we succeeded in obtaining a proof for the acceptable set and designing an iterative optimization method for an IMRT treatment planning including dose-volume constraints.

## Figures and Tables

**Figure 1:** Schematic diagram of strategy for searching for nearly optimal solution.

**Figure 2:** Phantom images of (a) C-shape for acceptable planning and (b) extended C-shape simulating the head and neck for remaining-one unacceptable planning. The red region shows PTV, and the blue and green regions indicate OARs.

**Figure 3:** DVH of (a) PTV with (*K*_1_, *b*_1_^*U*^, *ζ*_1_^*U*^) and (*K*_1_, *b*_1_^*L*^, *ζ*_1_^*L*^) and (b) OAR with (*K*_2_, *b*_2_^*U*^, *ζ*_2_^*U*^) obtained for acceptable planning. The red right-angle corners indicate DVCs in Table 1.

**Figure 4:** Time evolution of divergence *V* for acceptable planning.

**Figure 5:** Time evolutions of (a) ∣*ℐ*_1_^*U*^ | /*I*_1_ and *R*_1_^*U*^ , (b) ∣*ℐ*_1_^*L*^ | /*I*_1_ and *R*_1_^*L*^, and (c) ∣*ℐ*_2_^*U*^ | /*I*_2_ and *R*_2_^*U*^ for acceptable planning. A red line indicates the prescribed proportion rate.

**Figure 6:** DVH of (a) PTV with (*K*_1_, *b*_1_^*U*^, *ζ*_1_^*U*^) and (*K*_1_, *b*_1_^*L*^, *ζ*_1_^*L*^), (b) OAR (spinal cord) with (*K*_2_, *b*_2_^*U*^, *ζ*_2_^*U*^), and (c) OAR (parotid) with (*K*_3_, *b*_3_^*U*^, *ζ*_3_^*U*^) obtained for totally unacceptable planning. The red right-angle corners indicate DVCs in Table 2.

**Figure 7:** DVH of (a) PTV with (*K*_1_, *b*_1_^*U*^, *ζ*_1_^*U*^) and (*K*_1_, *b*_1_^*L*^, *ζ*_1_^*L*^), (b) OAR (spinal cord) with (*K*_2_, *b*_2_^*U*^, *ζ*_2_^*U*^), and (c) OAR (parotid) with (*K*_3_, *b*_3_^*U*^, *ζ*_3_^*U*^) obtained for partly acceptable planning. The red right-angle corners indicate DVCs in Table 2.

**Figure 8:** DVH of (a) PTV with (*K*_1_, *b*_1_^*U*^, *ζ*_1_^*U*^) and (*K*_1_, *b*_1_^*L*^, *ζ*_1_^*L*^), (b) OAR (spinal cord) with (*K*_2_, *b*_2_^*U*^, *ζ*_2_^*U*^), and (c) OAR (parotid) with (*K*_3_, *b*_3_^*U*^, *ζ*_3_^*U*^) obtained by the proposed procedure for remaining-one unacceptable planning. The red right-angle corners indicate DVCs in Table 2.

**Figure 9:** Time evolution of distances *U*_*e*_ (blue) and *U*_*r*_ (red) obtained using Procedure 7 for remaining-one unacceptable planning.

**Figure 10:** Relation between *λ* versus *U*_*r*_(*z*(*N*_1_ + *N*_2_)) (red dots) and *N*_2_ (green dots) on left and right axes, respectively.

**Table 1:** The prescribed constraints and equivalent parameters for acceptable planning (*V*_*d*_ denotes the percentage of volume receiving at least *d* [Gy]).

Assigned region (colored region in Figure 2(a))	Organ	Constraint	Equivalent parameter
PTV (red)	PTV	*V*_55_ < 10%	(*K*_1_, *b*_1_^*U*^, *ζ*_1_^*U*^) with *b*_1_^*U*^ = 55 and *ζ*_1_^*U*^ = 0.90
		*V*_50_ ≥ 95%	(*K*_1_, *b*_1_^*L*^, *ζ*_1_^*L*^) with *b*_1_^*L*^ = 50 and *ζ*_1_^*L*^ = 0.95

OAR (blue)	Core	*V*_10_ < 5%	(*K*_2_, *b*_2_^*U*^, *ζ*_2_^*U*^) with *b*_2_^*U*^ = 10 and *ζ*_2_^*U*^ = 0.95

**Table 2:** The prescribed constraints and equivalent parameters for partly unacceptable planning (*V*_*d*_ and *D*_mean_ denote the percentage of volume receiving at least *d* [Gy] and mean dose, respectively).

Assigned region (colored region in Figure 2(b))	Organ	Constraint	Equivalent parameter
PTV (red)	PTV	*V*_75_ < 5%	(*K*_1_, *b*_1_^*U*^, *ζ*_1_^*U*^) with *b*_1_^*U*^ = 75 and *ζ*_1_^*U*^ = 0.95
		*V*_70_ ≥ 95%	(*K*_1_, *b*_1_^*L*^, *ζ*_1_^*L*^) with *b*_1_^*L*^ = 70 and *ζ*_1_^*L*^ = 0.95

OAR (blue)	Spinal cord	*V*_30_ = 0%	(*K*_2_, *b*_2_^*U*^, *ζ*_2_^*U*^) with *b*_2_^*U*^ = 30 and *ζ*_2_^*U*^ = 1
		*D*_mean_ ≤ 10 Gy	(*K*_2_, *c*_2_^*U*^) with *c*_2_^*U*^ = 10

OAR (green)	Parotid	*V*_5_ < 50%	(*K*_3_, *b*_3_^*U*^, *ζ*_3_^*U*^) with *b*_3_^*U*^ = 5 and *ζ*_3_^*U*^ = 0.5
		*D*_mean_ ≤ 10 Gy	(*K*_3_, *c*_3_^*U*^) with *c*_3_^*U*^ = 10

## Data Availability

All data used to support the findings of this study are included within the paper.
